The article "Predicting the Risk of Depression Based on ECG Using RNN" was retracted in 2023. Reasons: signs of a paper mill; compromised peer review; unreliable results or conclusions.

# Predicting the Risk of Depression Based on ECG Using RNN

**DOI:** 10.1155/2021/1299870

**Published:** 2021-07-28

**Authors:** Sumaiya Tarannum Noor, Syeda Tasmiah Asad, Mohammad Monirujjaman Khan, Gurjot Singh Gaba, Jehad F. Al-Amri, Mehedi Masud

**Affiliations:** ^1^Department of Electrical and Computer Engineering, North South University, Bashundhara, Dhaka 1229, Bangladesh; ^2^School of Electronics and Electrical Engineering, Lovely Professional University, Phagwara, India; ^3^Department of Information Technology, College of Computers and Information Technology, Taif University, P. O. Box 11099, Taif 21944, Saudi Arabia; ^4^Department of Computer Science, College of Computers and Information Technology, Taif University, P. O. Box 11099, Taif 21944, Saudi Arabia

## Abstract

This paper presents a model to predict the risk of depression based on electrocardiogram (ECG). This proposed model uses a Recurrent Neural Network (RNN) and Long Short-Term Memory (LSTM) autoencoder to predict normal, abnormal, and PVC heartbeats. The RNN model is a deep learning-based model to classify normal, abnormal, and PVC heartbeats. We used the model as a classifier. The model uses a heart rates dataset to predict abnormal and PVC heartbeats. As for the dataset, we have used 5000 ECG samples. The model was trained on a training dataset and validation dataset. After that, it was tested on a test dataset. The model is trained on normal heartbeat rates, so the model can predict any heartbeat rates other than normal. Our contribution here is to build a model that can differentiate between “normal,” “abnormal,” and “risky” heartbeats. Our model predicts “normal” heartbeats with 97.24% accuracy and can predict “PVC” heartbeats with 100% accuracy. Other than the accuracy, we evaluated our model on the training loss graphs. These two types of training loss graphs were evaluated as “normal” versus “risky” and “abnormal” versus “risky.” We have seen great results there as well. The best losses for “normal,” “abnormal,” and “risky” are 5.71, 33.36, and 34.78. However, these results may improve if a larger dataset is used. In studies, it was found that patients suffering from depression may have a different kind of heartbeat than the normal ones. In most cases, it is PVC (Premature Ventricular Contraction) heartbeats. Therefore, the target is to predict abnormal heartbeats and PVC heartbeats.

## 1. Introduction

ECG is a painless and common process. This ECG is basically a graph of voltage versus time. The heart's electric activity is shown in the graph, which is collected using an electrode placed on the skin. These electrodes are conductive pads that are attached to the body. Approximately 10 electrodes with adhesive are attached to the skin of your chest, arm, and legs. Many common heart problems are predicted through ECG. It is used to predict abnormal heart rhythm (arrhythmia), blocked or narrowed arteries in the heart caused by “coronary artery disease” that may cause chest pain or heart attack, the possibility of a previous heart attack, and functioning of a pacemaker. Heartbeat rate is the number of pulses a heart makes per minute. Heartbeat rate is directly connected to our health. While the heart beats, blood containing oxygen and nutrients circulate through our body. The heartbeat rate goes higher if one gets involved in the exercise. There are two types of heartbeat rates: target heartbeat rate and maximum heartbeat rate. Through many studies [1–3], the authors took 75–100 the normal heartbeat rate of an adult. If the heart starts to beat in an irregular system, it can be considered an abnormal heart rate. R-on-T Premature Ventricular Contraction (R-on-T PVC) is caused by a ventricular ectopic focus (abnormal pacemaker sites within the heart). It produces an early and broad QRS complex (a combination of *Q* wave, *R* wave, and S wave). PVC is called premature because it occurs before a heartbeat, Supraventricular Premature, or Ectopic Beat (SP or EB). It is a kind of heartbeat rate that is caused by atrial contraction that is triggered by ectopic foci. All these abnormal heart conditions can lead to a heartbeat rate that is not within the range of 75–100 bpm.

The article "Predicting the Risk of Depression Based on ECG Using RNN" was retracted in 2023. Reasons: signs of a paper mill; compromised peer review; unreliable results or conclusions.

RNN is a kind of deep learning model architecture. It is a class of artificial neural networks. In RNN, the layers are connected so that the recurrent process can take place. Here, the outputs of a layer can be fed to any previous layer so that the model can get well trained. It uses the concept of memory and a feed-forward neural network. For these, RNN is able to recognize patterns. RNNs are divided into four categories: one-to-one, one-to-many, many-to-one, and many-to-many. LSTM is a form of RNN that can learn long-term relationships. LSTM is used for different kinds of recognition-related tasks, such as handwriting recognition and speech recognition.

We built an RNN model that is a simpler approach to neural network, which also includes an LSTM autoencoder. We took a simpler approach than CNN. Our model can work with ECG datasets. For our model, we have used the time series of the ECG datasets. We used 3 layers of encoder and decoder in the LSTM autoencoder and trained the model for 150 epochs. We got an accuracy of 97.24% while predicting “normal” heartbeats and 100% accuracy while predicting “PVC” or “risky” heartbeats. These results can be improved if we use a bigger time-series dataset of ECGs.

The article "Predicting the Risk of Depression Based on ECG Using RNN" was retracted in 2023. Reasons: signs of a paper mill; compromised peer review; unreliable results or conclusions.

## 2. Related Works

Deep learning and machine learning models are widely used for medical diagnosis [4–7]. We now discuss the related works related to predict the risk of depression.

### 2.1. Discussion of the Studies Based on “Depression” and Its Risks

In different studies [8–10], it is shown that in patients who are suffering from “depression,” it is seen that their heartbeat rate is not normal. Depression leads to some major problems; that is, it affects the heart and its performance, leads to an unhealthy lifestyle, may lead the patient to commit suicide, or may lead to self-harming activities which can make a patient a drug addict. The authors intend to predict depression so that perfect medication can be given at the right time. In [11, 12], studies show that depression can affect the mortality rate.

### 2.2. Discussion of Related Works

To diagnose depression using electroencephalogram (EEG) signals, the author constructed a hybrid model employing Convolution Neural Network (CNN) and LSTM architectures in [13]. CNN layers learn the signals, and LSTM layers give the sequence learning mechanism in the model. EEG signals from the left and right hemispheres of the brain are collected here. This model recognizes depression using EEG signals much more quickly. In [14], the author analyzes several ECG signals and determines the person's state of depression. To predict problems in the heart, this model included a feature extraction algorithm. A web application was also developed to extract attributes of ECG signals such as the ST segment and QRS wave, utilizing these characteristics to show whether one is suffering from hyperacute stress (myocardial infarction), acute stress (Type A), hyperchronic stress (ischemia), or chronic stress (Type B). In [15], the author proposed a process that identifies aberrant signals in cardiovascular patients' ECGs. To determine ST depression from aberrant ECG data, an appropriate correlation coefficient threshold was chosen. Furthermore, a cross-validation approach that is based on a correlation coefficient between the ECG data on the pattern in ST depression and other disorders was employed to define an optimal threshold in this system. These findings can be used to optimize the use of smartphones or tablets in online research by reducing calculating time.

In [16], the author has introduced a machine learning-based model and automated prediction of depression model using linear and nonlinear HRV measures and using a categorization and characteristic assortment method. A support vector machine-recursive feature elimination (SVM-RFE) and a statistical filter were utilized as classification algorithms. Twenty HRV plots were generated from ECG recordings, with 13 linear, five nonlinear, and two Poincare plots. In [17], the author developed a model using the actual ECG records to notice irregularities in a patient's heartbeat. An LSTM autoencoder is used to predict those anomalies. After that, the model was trained on regular heartbeats and classified unnoticed models as regular or anomalies.

The article "Predicting the Risk of Depression Based on ECG Using RNN" was retracted in 2023. Reasons: signs of a paper mill; compromised peer review; unreliable results or conclusions.

### 2.3. Our Contribution

The existing systems have used ECG datasets [14–16]. But some of them have used CNN. Here, in this system, the ECG heartbeat rate data is used as the dataset. To build the model, an RNN with an LSTM autoencoder is used. The main differences between our system and the existing ones are the dataset and the neural network model. As the previous systems had already used CNN, we decided to use RNN for the model. Also, we decided to use ECG heartbeat rates other than the EEG dataset to train our model. Our main contribution here is that we have built a model that is a simpler approach to neural networks, that is, RNN, which also includes an LSTM autoencoder. Another contribution is that our model can work with ECG datasets, which are a valuable resource while predicting different types of diseases.

### 2.4. Comparison between Related Works and Our Contribution

Table 1 shows the comparison results of the related works and the proposed model.

### 2.5. Advantages and Disadvantages of Our Model

Our model uses Recurrent Neural Network (RNN). This approach is easier than Convolutional Neural Network (CNN). So, our model is much simpler than most of the existing models. We have also included the LSTM autoencoder to make our model perform better. We used 3 layers in both the encoder and decoder; therefore, the performance is good. There is no particular disadvantage to our model. We can say a limitation may be that it works for the time-series dataset.

## 3. Methods and Methodology

In this section, the authors present the diagrams: block, architectural, and LSTM diagrams and all the processes for each part. Other than the diagrams, the rest are developed using “PyTorch.” The authors of this paper have taken references and help from [17].

### 3.1. Outline of the Full System Using Block Diagram

The system is depicted in Figure 1 as a block diagram. In the block diagram, the whole process of the model is shown in detail. First of all, the model takes raw ECG signals from a dataset, which is real-world ECG data. The RNN learns the signals from the dataset and passes those signals to the LSTM autoencoder. There are two parts to the autoencoder architecture in common. The encoder compresses the input, the decoder attempts to recreate it, and the recurrent autoencoder joins the encoder and decoder, capturing the regenerated ECG signals. The training process is done based on those signals. A threshold value has been taken to predict normal and risky heartbeat. After comparing normal and risky heartbeat, the models record the prediction between normal and risky and abnormal and risky (PVC).

The article "Predicting the Risk of Depression Based on ECG Using RNN" was retracted in 2023. Reasons: signs of a paper mill; compromised peer review; unreliable results or conclusions.

### 3.2. Architecture of the Whole System (Deep Learning Model-RNN)

Figure 2 shows the architecture diagram of the system. In the architecture of the system, where the model gets input from the dataset. After that, the data preprocessing has been done to rename some columns in the dataset, and the data exploration has been done to explore the dataset. Then, RNN learns those data and sends them to the LSTM autoencoder for model training. After completing the training process, the testing part is done on training data to classify and predict normal and risky heartbeats. This is how this model gets the predicted output.

There are two parts to the standard autoencoder structure. An encoder compresses the input, while a decoder attempts to recreate it, and then those reconstructed input values will give us the output predictions [18].

### 3.3. Architecture of the LSTM Autoencoder

The autoencoder's task is to receive some input data, run this through the system, and recreate the input.  Figure 3 shows the architecture diagram of the LSTM autoencoder. As much as possible, the recreation should resemble the input. In this model, the encoder uses three LSTM layers to compress the data input and decodes the compressed representation using a decoder. The decoder also contains three LSTM layers, and an output layer that provides the ultimate reconstruction [19].

### 3.4. Data, Data Exploration, and Data Preprocessing

This research considered the data from [20]. The dataset is a time-series dataset. It includes the ECG heartbeat rates in a time-series manner. This dataset contains the heartbeat rates for 5000 patients that contain 140 timesteps. There are five types of heartbeat rates that include normal (N), R-on-T Premature Ventricular Contraction (R-ONT PVC), Premature Ventricular Contraction (PVC), Supraventricular Premature or Ectopic Beat (SP or BP), and Unclassified Beat (UB).

The dataset was downloaded and unzipped for use. The dataset came in “arff” format. As the dataset was previously parted into “train-size”  =  500 and “test-size”  =   4500, it was combined to be used in a better way. After that, its shape was defined, which is (5000, 141). Possible classes were named. Both “normal” and “PVC” were defined separately as later work will be done with these two. The authors of this paper took PVC as the “risky” heartbeat at the end where the comparison graph will be shown but did not name the class as “risky” for the sake of code accuracy. Therefore, in the rest of the paper, in most cases, it is defined as a “PVC” heartbeat.

The article "Predicting the Risk of Depression Based on ECG Using RNN" was retracted in 2023. Reasons: signs of a paper mill; compromised peer review; unreliable results or conclusions.

The dataset values are processed in the data preprocessing part and shown in 5 rows *x* 141 columns. In the data exploration part, the dataset classes are plotted and shown in Figure 4.

From Figure 4, it is clear that both “normal” and “PVC” have the most examples.

### 3.5. Time-Series Graph for Each Class

In this part, the time series for each class is shown in Figure 5. These are the graphs that show how each heartbeat's time-series graphs should look like. These figures only show the graphs for our dataset, which contains 5000 ECG samples. For a bigger dataset, these graphs may contain more maximum and minimum points. So, it would be much easier to differentiate the “normal” heartbeat.

From Figure 5, it is clearly seen that “normal” heartbeats have a much different curve than others, which can surely give benefits while comparing among them. Though the “PVC” class is quite similar to “R-on-T,” “SP,” and “UB”; still, it is quite different looking and will help while comparing.

### 3.6. Shapes of Important Classes

In this part, the authors of this paper have shown the shapes for important classes. For the “normal” class, the shape is (2919, 140). All the classes that are not “normal” classes are classified as “abnormal” classes. It has got a shape of (2081, 140). The “PVC” heartbeat class is showing a shape of (1767, 140). It is showing 140 for the column shape as the “target” class was dropped.

### 3.7. Tensor Creation from the Dataset

The authors created tensors from example classes to use them further in the system for training and testing. Here, three types of tensors are created for testing: normal, abnormal, and PVC. All of these datasets are 2D tensors. They have a sequence length of 140 and have only one feature.  Table 2 shows the tensor list from the dataset.

### 3.8. Autoencoder

The system uses an LSTM Autoencoder. This autoencoder has two parts: encoder and decoder. The encoder part uses three LSTM layers to compress the data. This way, the encoder encodes the data to be used in its lowest dimension. After that, the dataset enters into the decoder part. The decoder part also has three LSTM layers. Using these layers, the decoder reconstructs the dataset.

The recurrent autoencoder is the part where the RNN concept of deep learning is used. In this part, the data recurrently gets into the autoencoder for compression and reconstruction.

### 3.9. Training Process of the Model

The system was trained using 150 epochs. A training dataset and validation dataset were used while training to avoid overfitting. Throughout the training process of 150 epochs, our training loss and validation loss decreased gradually.  Table 3 provides the training parameters of the model.

The article "Predicting the Risk of Depression Based on ECG Using RNN" was retracted in 2023. Reasons: signs of a paper mill; compromised peer review; unreliable results or conclusions.

For the training process, the “L1Loss”function is used that measures MSE (mean squared error) and MAE (mean absolute error). It generates a standard that can measure the MAE (mean absolute error) between the input and the goal output. If the unreduced loss is considered as a function, it can be shown as a function.

If the “reduction” is set to “none,” then loss can be described as

(1) $$\begin{array}{c} L\left(x,y\right)=L={\left\{l_{1},\ldots ,\ldots ,\ldots ,l_{n}\right\}}^{T},\\ l_{n}=\left|x_{n}-y_{n}\right|. \end{array}$$

where *n*  =  is batch size.

If the “reduction” is not set to “none,” then loss can be described as

(2) $$\begin{array}{c} l\left(x,\;y\right)=\text{mean }\left(L\right)\text{,if reduction }=\;\prime \text{mean,}\\ l\left(x,\;y\right)=\text{sum }\left(L\right)\text{,if reduction }=\;\prime \text{sum.} \end{array}$$

At the 150^th^ epoch, the training loss is approximately 8.88, and the validation loss is approximately 9.59. As the validation loss is decreasing over time, the accuracy of the model increased. The training loss and validation loss are plotted into the “loss versus epoch” graph. The graph is shown in Figure 6.

From Figure 6, it can be seen that the training graph and the testing graph are quite similar. From here, it can be concluded that the model is quite accurate. It is neither overfitting nor underfitting. As Figure 6 shows a perfect balance of loss and epochs, we can say that the model's performance is good.

### 3.10. Comparison Using the Threshold Value

The authors here in [17] used a function that is used to set a threshold value for this system. A threshold value is used to differentiate the heartbeats. Therefore, a graph is plotted based on the function. It records the prediction and losses for each example.  Figure 7 shows the train dataset loss graph from each example.

From this graph, the threshold value is set to 30. Examples that are below threshold value losses are considered as “normal” heartbeat, and any example above it is considered as “abnormal” or “risky.”

## 4. Accuracy Checkup and Resultant Figures

In this section, the authors of this paper have shown the system's accuracy graphs and resultant figures. All the references for this part were taken from [17].

### 4.1. Normal Heartbeat Prediction

For “normal” heartbeats, the system's correct prediction is 141 out of 145. This dataset is new for the model in this situation. So, it is actually getting tested for the new dataset. Therefore, the accuracy is (141/145) ^*∗*^ 100  =  97.24%. Other than this accuracy, we can see the graphs of ‘normal' heartbeats. This graph shows that the “normal” heartbeat is lower than the threshold value. This prediction is shown in Figure 8.

The article "Predicting the Risk of Depression Based on ECG Using RNN" was retracted in 2023. Reasons: signs of a paper mill; compromised peer review; unreliable results or conclusions.

### 4.2. Risky Heartbeat Prediction

For “risky” heartbeats prediction, the dataset for PVC heartbeats is used. The system's correct prediction is 145 out of 145. Therefore, the accuracy is (145/145) ^*∗*^ 100  =  100%. This accuracy rate can decrease if a larger dataset is used. This graph shows the “risky” heartbeats. We can clearly see that they are all greater than the threshold value. This prediction is shown in Figure 9.

### 4.3. Time-Series Prediction: Normal versus Risky

In this section, the authors of this paper compared “normal” heartbeats and “risky” heartbeats. They are plotted and shown using a time series. For the “risky” heartbeats, the dataset for “PVC” heartbeats is used, as “PVC” heartbeat carries the risk of depression in patients. We have used training loss for this comparison. From this graph, we can see the best and worst training loss in these 12 examples. The comparison can be seen in Figure 10.

From Figure 10, it can be seen, the “normal” heartbeats have the lowest loss, 5.71, and the highest loss, 13.36, while the “risky” heartbeats have the lowest loss of 34.78 and the highest loss of 64.66. So, the heartbeats can easily be differentiated. Figure 10 clearly shows the differences of “normal” and “risky” heartbeats reconstructed graphs. So, we can easily predict them.

### 4.4. Time-Series Prediction: Abnormal versus Risky

In this section, the authors of this paper compared “abnormal” heartbeats and “risky” heartbeats. They are plotted and shown using a time series. For the “risky” heartbeats, the dataset for “PVC” heartbeats is used, as “PVC” heartbeat carries the risk of depression in patients. Abnormal heartbeats can lead to many other diseases, which are also detrimental. We have used the same approach as the previous section. The comparison can be seen in Figure 11.

From this image, it can be seen that the “abnormal” heartbeats have the lowest loss, 33.36, and the highest loss, 64.66, while the “risky” heartbeats have the lowest loss, 34.78, and the highest loss, 64.66. The heartbeats have similarities as the “abnormal” heartbeat class includes the “PVC” heartbeat class. Yet, they show many different values. Figure 11 clearly shows the differences between “normal” and “risky” heartbeats reconstructed graphs. So, we can easily predict them. If a bigger dataset is used, including many different examples, this system will be able to differentiate between them as well. Then, by looking at the time-series graph comparisons, normal heart disease and mental illness or depression prediction will be possible. As in [11, 12], it can be seen that depression can increase the mortality rate. Therefore, this prediction can lead to a long way toward better treatment for depression and may positively affect the mortality rate.

The article "Predicting the Risk of Depression Based on ECG Using RNN" was retracted in 2023. Reasons: signs of a paper mill; compromised peer review; unreliable results or conclusions.

### 4.5. Accuracy of the System

Table 4 presents the accuracy of the system. The table includes the accuracy of the best model and the best algorithm that has been used on this dataset and our model's accuracy.

From Table 4, we can clearly see the differences between the accuracies. The best algorithm and best model that was used for this dataset gave 94.61% accuracy [20], whereas our model gives 97.24% accuracy. Our model gives us better accuracy as we have used RNN and LSTM autoencoder. Its performance is better than the best model as we can see the difference. Therefore, it can be concluded that our model is working excellently.

## 5. Conclusion

The authors of this paper tried to find a solution to a real-life problem. The system can predict “normal” heartbeat with 97.24% accuracy, whereas the best model that has used this dataset gives 94.61% accuracy. Future work is possible in different sections of this system. A more extensive dataset that can provide a better training set and a validation set can be more useful. This model is much simpler than the other existing models, and the prediction results are praiseworthy. This model can be improved in the future using a better and bigger dataset and commercial funding. Therefore, it will become suitable to be used for medical-related purposes. Depression is a major cause that leads to an imbalanced way of life. It is hard to predict a depressed person. Therefore, using this system may pave a new path in the treatment process of “depression” and many other illnesses.

## Figures and Tables

**Figure 1:** Block diagram for the system.

**Figure 2:** Architecture diagram for the system.

**Figure 3:** Architecture diagram of the LSTM autoencoder.

**Figure 4:** Five types of heartbeat classes in the dataset.

**Figure 5:** Time series graph for each heartbeat class.

**Figure 6:** Loss versus epoch graph.

**Figure 7:** Train dataset loss graph from each example.

**Figure 8:** Normal heartbeat dataset loss that is under the threshold value.

**Figure 9:** “PVC” or “risky” heartbeat dataset loss that are over the threshold value.

**Figure 10:** Overlapping graph of “true” and “reconstructed” time-series graph of “normal” and “PVC”/”risky” heartbeat.

**Figure 11:** Overlapping graph of “true” and “reconstructed” time-series graph of “abnormal” and “PVC”/”risky” heartbeat.

The article "Predicting the Risk of Depression Based on ECG Using RNN" was retracted in 2023. Reasons: signs of a paper mill; compromised peer review; unreliable results or conclusions.

**Table 1:** Comparison table.

Related works	Their model	Accuracy	Our model
In [13]	CNN and LSTM architecture	97.66–99.12%	**—**
In [14]	Feature extraction algorithm	Not mentioned	
In [15]	Cross validation	90–97%	
In [16]	Machine learning model	74.4%	
In [17]	LSTM autoencoder	Not mentioned	
	RNN and LSTM autoencoder	97.24%	

**Table 2:** Tensor list from the dataset.

Dataset	Number of images
Training	1401
Validation	963
Testing	438

**Table 3:** Training parameters of the model.

Parameters	Value
Learn rate	0.001
Best loss	10000.0
Batch size	1
Optimization algorithm	Adam
Number of epochs	150
Execution environment	GPU

**Table 4:** Model comparison in terms of accuracy.

Best algorithm model	Our model (%)
94.61% [20]	97.24

## Data Availability

The data used to support the findings of this study are freely available at http://timeseriesclassification.com/description.php?Dataset=ECG5000.
